RETRACTED

# Analyzing the regional economic changes in a high-tech industrial development zone using machine learning algorithms

**DOI:** 10.1371/journal.pone.0250802

**Published:** 2021-06-22

**Authors:** ErLe Du, Meng Ji

**Affiliations:** Department of Strategic Development, Harbin Bank, Harbin, China; Qingdao University, CHINA

## Abstract

The aims are to improve the efficiency in analyzing the regional economic changes in China’s high-tech industrial development zones (IDZs), ensure the industrial structural integrity, and comprehensively understand the roles of capital, technology, and talents in regional economic structural changes. According to previous works, the economic efficiency and impact mechanism of China’s high-tech IDZ are analyzed profoundly. The machine learning (ML)-based Data Envelopment Analysis (DEA) and Malmquist index measurement algorithms are adopted to analyze the dynamic and static characteristics of high-tech IDZ’s economic data from 2009 to 2019. Furthermore, a high-tech IDZ economic efficiency influencing factor model is built. Based on the detailed data of a high-tech IDZ, the regional economic changes are analyzed from the following dimensions: economic environment, economic structure, number of talents, capital investment, and high-tech IDZ’s regional scale, which verifies the effectiveness of the proposed model further. Results demonstrate that the comprehensive economic efficiency of all national high-tech IDZs in China is relatively high. However, there are huge differences among different regions. The economic efficiency of the eastern region is significantly lower than the national average. The economic structure, number of talents, capital investment, and economic efficiency of the high-tech IDZs show a significant positive correlation. The economic changes in high-tech IDZs can be improved through the secondary industry, employee value, and funding input. The ML technology applied can make data processing more efficient, providing proper suggestions for developing China’s high-tech industrial parks.

## Introduction

The high-tech industrial development zone (IDZ) is a vital measure promoted by Chinese policy, aiming to improve enterprises’ innovation capabilities and find the driving force for new economic development [1]. In the past decade, the average annual growth rate of China’s high-tech industry’s overall annual output value was 23.15%, and the growth rate of fixed assets was 18.19%. Hence, the impact of high-tech industries on China’s economic development is notable [2]. Due to the economic differences of different regions in China, different high-tech IDZs have different development directions. Guangdong Province’s high-tech industry’s total output value is more than twice the sum of the entire central and western regions. This unbalanced development has restricted the development of China’s high-tech industry [3]. Under the reasonable guidance of national policies, different regions take their local economic development into considerations, focusing on the introduction of characteristic industries and circular economy. Only in this way can the high-tech industries in different regions expand.

RETRACTED

Moreover, the professional orientation of each high-tech IDZ becomes more prominent, which significantly promotes the development of China’s independent innovation industry, providing an impetus for innovation-driven development [4]. Recently, under the downward pressure of the international and Chinese economies, the resistance to high-tech industries’ development has also increased. Although some regions have similar development processes to those of other regions, the speed of economic development and economic efficiency are quite different [5]. Therefore, studying the regional economic changes of high-tech IDZs, understanding the factors that influence the development of high-tech industries, and truly realizing the transformation and development of high-tech industries are vital for China’s economic development.

With the rapid development of the internet economy, more fields and areas have adopted information technology to improve data processing efficiency [6]. Scholars also utilize machine learning (ML) algorithm to solve the problems effectively in the economic field. Vilar et al. (2016) employed the Generalized Linear Model (GLM) and the ML Maximum Entropy (Maxent) model to predict fire hazards in the 1980s and 2000s, in an effort to identify the changes in the socio-economic driving factors that affected the fire hazards in each period. Results found that the model could be effectively modeled [7]. Nosratabadi et al. (2020) adopted four separate categories of deep learning models, hybrid deep learning models, hybrid ML, and integrated models to analyze economic data and found that the hybrid model performed better than other learning algorithms [8]. Ghoddusi et al. (2019) found that Support Vector Machine (SVM), Artificial Neural Network (ANN), and Genetic Algorithm (GA) were the most widely used models in the economic field, providing research ideas for the fields of energy economics and finance [9]. Storm et al. (2020) believed that when economists adopt quantitative analysis to solve economic problems, the ML approach should be the top priority, which could quickly and efficiently solve economic problems [10]. Hence, ML is effectively applied in the economic field and can improve forecasting efficiency and accuracy. However, there are few specific practical ML applications in this field; ML methods have not been implemented at the actual implementation level.

RETRACTED

Therefore, in response to the above problems, the ML algorithms are adopted to establish a regional economic analysis model based on previous works. The model uses data envelopment analysis (DEA) and Malmquist index measurement algorithms to analyze the economic data in a high-tech IDZ from 2010–2019. The regional economic changes are analyzed from the following dimensions: economic environment, economic structure, number of talents, capital investment, and high-tech IDZ’s regional scale. Also, high-tech industrial development and its influence mechanism are analyzed as well. The results can provide a theoretical basis for the government and economic investment institutions.

High-tech IDZs can be better developed under the support of a sound business environment, preferential policies, and optimized resource allocation. The analysis and research of economic efficiency will help understand the resource utilization in different high-tech IDZs, formulate favorable policies, and make full use of resources available, thereby enhancing the competitiveness of high-tech IDZs and gaining competitive advantages under the market economy. Therefore, the understanding of the impact mechanism of the economic efficiency of high-tech IDZs is deepened through the empirical efficiency analysis and research on influencing factors, which can help reveal the reasons for the efficiency differences of high-tech IDZs and put forward suggestions. Hopefully, high-tech IDZs in backward areas can be promoted, China’s high-tech IDZs can be developed comprehensively and healthily, and the economic efficiency can be improved, which is of practical significance in promoting economic transformation and achieving rapid economic development.

## Materials and methods

### Traditional regional economic analysis

The traditional regional economic analysis mainly adopts the Data Envelopment Analysis (DEA) model [11], which calculates relative efficiency by calculating the economic efficiency between different departments. This model is often combined with the Banker-Charnes-Cooper (BCC) model. It assumes the Differential Unitary Modulation (DMU) in the case of variable returning to scale, thereby analyzing the pure technology and scale efficiency. This model measures the efficiency of departments with multiple inputs and multiple outputs [12]. The traditional DEA model can set different guidance parameters according to the measurement goal. The guidance under the BCC model can be expressed as:

$$\min\theta -\varepsilon (e^{T}S^{-}+e^{T}S^{+})$$ (1)

$$s.t.\{\begin{array}{l} \sum_{j=1}^{n}X_{j}\lambda_{j}+S^{-}=\theta X_{0}\\ \sum_{j=1}^{n}Y_{j}\lambda_{j}-S^{+}=Y_{0}\\ \lambda_{j}\geq 0,S^{-},S^{+}\geq 0 \end{array}$$ (2)

In (1) and (2), *j = 112*, *…*, *n* represents decision-making units (DMUs), *X* represents the input vector, and *Y* stands for the output vector. The efficiency value calculated by the BCC model is the comprehensive technical efficiency (TE), which can be decomposed into the scale efficiency (SE) and the pure technical efficiency (PTE), where:

TE=SE*PTE (3)

This method can effectively analyze and process the economic efficiency of different regions and different times. However, the model has limitations. When multiple DUMs appear, the efficiency will always be 1, making it impossible to compare the efficiency of different samples; hence, this method has particular limitations [13].

RETRACTED

### ML super efficiency algorithm

The super efficiency algorithm is in the DUM operation, and the efficiency is not calculated in the system. Compared with other DUMs, the calculation result of super efficiency will generally be greater than 1 so that different samples can be compared and analyzed. Fig 1 illustrates the principles of the algorithm [14]. In Fig 1, DMU1, DMU2, and DMU3 constitute three useful DMU points. When studying the super efficiency of DMU2, point DMU2 is excluded from the efficiency frontier. At this moment, the efficiency frontier consists of DMU1 and DMU3. The projection of point DMU2 on DMU1 and DUM3 is B, which reflects the excess efficiency of DMU2, i.e., its super efficiency value [15]. The calculation and qualification conditions are:

minθ (4)

$$s.t.\{\begin{array}{l} \sum_{j=1,j\neq k}^{n}\lambda_{j}X_{ij}\leq \theta X_{0}\\ \sum_{j=1}^{n}\lambda_{j}Y_{rj}\geq Y_{rk}\\ \lambda \geq 0,i=1.2,\ldots ,q,r=1,2,..,q,j=1,2,\ldots n \end{array}$$ (5)

**Fig 1:** Structure of super efficiency principles.

### ML Malmquist algorithm

Malmquist is an algorithm that analyzes the dynamic changes between output and input. Since the algorithm does not require specific input and output prices, it does not need to make assumptions about the research sample. Therefore, it is often used to evaluate and analyze economic data [16]. The equation is the geometric average of the period *t* to *t+1*. Compared with other algorithms, this model can analyze the regional economic efficiency changes in different high-tech IDZs according to particular time changes, without the necessity to set specific functions; besides, the data are relatively easy to obtain [17]. The specific equation is as follows:

$$M_{0}(X^{t+1},Y^{t+1},X_{t},Y_{t})=[\frac{D_{0}^{t+1}(X^{t+1},Y^{t+1}|CRS)D_{0}^{t}(X^{t+1},Y^{t+1}|CRS)}{D_{0}^{t+1}(X^{t},Y^{t}|CRS)D_{0}^{t}(X^{t},Y^{t}|CRS)}]$$ (6)

In (6), $D_{0}^{t}(X^{t},Y^{t})$ to $D_{0}^{t+1}(X^{t+1},Y^{t+1})$ represent the single-period output difference, and $D_{0}^{t+1}(X^{t+1},Y^{t+1})$ to $D_{0}^{t}(X^{t+1},Y^{t+1})$ represent the inter-period output difference. If *M*_0_(*X*^*t*+1^,*Y*^*t*+1^,*X*_*t*_,*Y*_*t*_)≥1 indicates that the production efficiency of the sample selected for empirical analysis has increased, then *M*_0_(*X*^*t*+1^,*Y*^*t*+1^,*X*_*t*_,*Y*_*t*_)≤1 indicates that the production efficiency has decreased. The Malmquist productivity index can be decomposed into the product of complete TE change and technical change (TC):

$$\begin{array}{l} M_{0}(X^{t+1},Y^{t+1},X_{t},Y_{t})=\frac{D_{0}^{t+1}(X^{t+1},Y^{t+1}|CRS)}{D_{0}^{t}(X^{t},Y^{t}|CRS)}\\ \left[\frac{D_{0}^{t+1}(X^{t+1},Y^{t+1}|CRS)D_{0}^{t}(X^{t+1},Y^{t+1}|CRS)}{D_{0}^{t}(X^{t},Y^{t}|CRS)D_{0}^{t+1}(X^{t},Y^{t}|CRS)}\right] \end{array}$$ (7)

Then, it is translated into complete TE changes:

$$EC(CRS)=\frac{D_{0}^{t+1}(X^{t+1},Y^{t+1}|CRS)}{D_{0}^{t}(X^{t},Y^{t}|CRS)}$$ (8)

$$TC(CRS)={\left[\frac{D_{0}^{t+1}(X^{t+1},Y^{t+1}|CRS)D_{0}^{t}(X^{t+1},Y^{t+1}|CRS)}{D_{0}^{t}(X^{t},Y^{t}|CRS)D_{0}^{t+1}(X^{t},Y^{t}|CRS)}\right]}^{1/2}$$ (9)

Efficiency changes (EC) indicate changes in overall TE. This value can reflect the management efficiency of high-tech IDZs and the impact on economic changes. If EC is greater than 1, then TE will be improved; on the contrary, if the value is less than 1, then TE will degrade [18]. TC reflect technological changes. A TC value greater than 1 represents technological progress, and vice versa [19].

RETRACTED

### Factor selection based on ML economic model

The key to measuring the economic efficiency of high-tech IDZs lies in selecting input indexes and output indexes. Under the DEA model, different indexes set for the same sample unit will significantly impact efficiency measurement, resulting in entirely different results. Moreover, they may even violate economic laws. Therefore, the selection of input and output indexes will be the emphasis. According to previous studies, the factors that affect economic efficiency are sorted out [20, 21]. Besides, based on the characteristics of China’s high-tech IDZs, five aspects are selected: economic environment, economic structure, number of talents, high-tech IDZ’s regional scale, and capital investment. The model construction is described, and the specific indexes and detailed explanations are shown in Table 1.

1. Economic environment: the average per capita income is selected to reflect the economic environment of high-tech IDZ. The average per capita income is significant to the efficiency of industrial development [22]. Therefore, it is assumed that the higher the average per capita income, the more conducive the environment is for the economic development of the high-tech IDZ, and the higher the economic efficiency of the high-tech IDZ.
2. Economic structure: the proportion of the secondary industry is selected, which reflects the economic situation of a region. At present, most Chinese regions’ secondary industry accounts for the majority, which is the primary driving force of China’s economic growth. Besides, the proportion of the secondary industry is also crucial to high-tech IDZ [23]. Therefore, it is assumed that the higher the proportion of the secondary industry in Gross Domestic Product (GDP), the higher the economic efficiency of the high-tech IDZ.
3. Number of talents: talents often determine the development level of different cities, having a positive correlation with economic efficiency. The importance of talents is vital in the era of national entrepreneurship. For high-tech IDZs, the talent competition is fiercer. The core of high-tech industries’ development is talents, which determine the pace of future industrial development [24]. Therefore, the number of talents is selected to measure the future development trend of high-tech IDZ. It is assumed that the more talents with senior titles in high-tech IDZ, the higher the high-tech IDZ’s regional efficiency.
4. High-tech IDZ’s regional scale: the high-tech IDZ’s regional scale here reflects the economic strength of a region and is the key to measuring the management level. As far as high-tech IDZ is concerned, the number and quality of enterprises are often affected by the infrastructure construction in the region, which will affect the economic efficiency of the industry [25]. Therefore, it is assumed that the larger the region, the higher its regional efficiency.
5. Capital investment: capital investment is the most important for high-tech IDZs, which mainly lies in whether the capital investment is used in actual research [26]. Therefore, annual statistical expenditures are utilized as an index. It is assumed that the greater the intensity of expenditures for high-tech IDZ, the higher its regional efficiency.

RETRACTED

**Table 1:** Variable selection of high-tech IDZ economic efficiency influencing factors.

Variable name	Variable connotation and calculation method
F1—Economic environment	Reflecting the overall economic environment factors of the city where the high-tech IDZ is located. The specific calculation is expressed in terms of GDP per capita.
F2—Economic structure	Reflecting the level of economic development of the high-tech IDZ and its knowledge and technological innovation capabilities. The specific calculation is expressed by the proportion of the secondary industry in GDP.
F3—Number of talents	Reflecting the endowment level of talent elements in the high-tech IDZ. The specific calculation is expressed by the proportion of personnel with intermediate and senior titles.
F4—High-tech IDZ’s regional scale	Reflecting the overall strength of the high-tech IDZ. It measures the management level of high-tech IDZ. The specific calculation is expressed by the proportion of the number of high-tech enterprises.
F5—Capital investment	Reflecting the economic strength of the high-tech IDZ and its emphasis on technological research and development. The specific calculation is expressed by the ratio of research and development expenditure to its technical income.

The above indexes are tested for correlation, and the calculation is as follows:

$$p(x,y)=\frac{\sum \left(x-\bar{x})(y-\bar{y}\right)}{\sqrt{\sum {\left(x-\bar{x}\right)}^{2}{\left(y-\bar{y}\right)}^{2}}}$$ (10)

Experiments prove that the correlation coefficients of all indexes are greater than ±0.1. Therefore, the selected variables are reasonable and can be used for subsequent analysis and modeling.

### Economic model construction based on ML

The high-tech IDZ comprehensive efficiency is taken as the dependent variable and other influencing factors as independent variables to construct a regression model for economic efficiency analysis of high-tech IDZ. According to the regression model, the overall efficiency value is a censored data y* between 0–1, y* is relevant to the regression factor, and the linear regression model is as follows:

$$y*=\alpha_{0}+\beta_{1}x_{i}+e_{i}\;i=1,2,\ldots ,n$$ (11)

In (11), y* is the censored data of the dependent variable, *α*_0_ is the constant term, *β*_1_ is the explanatory variable coefficient, *x*_*i*_ is the explanatory variable, and *e*_*i*_ is the disturbance term. The comprehensive efficiency of 20 high-tech IDZs is selected as the explained variable, denoted by *E*_*it*_; that is, the comprehensive efficiency of the *i*-th high-tech IDZ in the *t* period. According to the previous assumptions, five indexes, including economic environment, economic structure, number of talents, high-tech IDZ’s regional scale, and capital investment, are selected as explanatory variables, denoted as *F*_*1*_, *F*_*2*_, *F*_*3*_, *F*_*4*_, and *F*_*5*_. Here, the total efficiency values of 20 high-tech IDZs obtained from 2010 to 2019 are used as the explained variables. Based on the selected variables, the following model is established:

$$E_{it}=\alpha_{0}+\alpha_{1}F_{1\mathrm{it}}+\alpha_{2}F_{2\mathrm{it}}+\alpha_{3}F_{3\mathrm{it}}+\alpha_{4}F_{4\mathrm{it}}+\alpha_{5}F_{5\mathrm{it}}+e_{it}$$ (12)

The data used come from *China Statistical Yearbook 2010–2019* and *China Municipal Statistical Yearbook 2010–2019*. Some of the missing data are supplemented through the average method [27] to obtain a complete data analysis model. The specific selected high-tech IDZs are shown in Table 2. The detailed analysis process is presented in Fig 2.

RETRACTED

**Fig 2:** Operation flowchart of the system model.

**Table 2:** Selected city samples of high-tech IDZs.

Area classification	Variable connotation and calculation method
Northern region	B1—Beijing, B2—Tianjin, B3—Shijiazhuang, B4—Taiyuan
Southern region	C1—Fuzhou, C2—Xiamen, C3—Shenzhen, C4—Changsha
Eastern region	D1—Hangzhou, D2—Jiangsu, D3—Nanjing, D4—Hefei
Western region	E1—Xi’an, E2—Lanzhou, E3—Urumqi, E4—Luoyang

## Results and discussion

### Descriptive statistics

Fig 3 shows the descriptive statistics of each variable. The average value of all high-tech IDZ assets at the end of the year is 246.39 billion CNY. The year-end assets of each high-tech IDZ are quite different. The average value of high-tech IDZs’ actual use of technological activities is 52.88 billion CNY. The average number of employees is 157,920. The total income of each high-tech IDZ, total industrial output value, foreign exchange earnings from exports, and the number of employees vary greatly.

**Fig 3:** Descriptive statistics of each variable.

Fig 4 shows the descriptive statistics of comprehensive efficiency and influencing factors. The average efficiency of high-tech IDZs has reached 0.73, indicating that these five variables significantly impact the economy. Overall, the highest efficiency value is 1, and the lowest is 0.23. The economic efficiency value of high-tech IDZ varies greatly. The average value of the economic environment is 6,6678.7 CNY, the maximum is 19,017 CNY, and the minimum is only 12,978 CNY. The average value of the economic structure is 48.75, the maximum value is 85.08, and the minimum value is 18.57. The average value of the number of talents is 0.12, and the maximum value is 0.42. In other words, nearly half of the talents working in high-tech IDZs have intermediate and senior titles, and the minimum value is only 0.01. The average value of the high-tech IDZ’s regional scale is 0.38, of which the minimum is 0.02 and the maximum is 0.75. The average value of the capital investment in science and technology is 0.02, of which the minimum is 0.01, and the maximum is 0.05. The descriptive analysis of the data suggests that all variables show significant differences.

RETRACTED

**Fig 4:** Descriptive statistics of comprehensive efficiency and influencing factors. Note: In Fig 4, F1 to F5 respectively represent the economic environment, economic structure, number of talents, high-tech IDZ’s regional scale, capital investment, and comprehensive efficiency.

Fig 5 shows the regression analysis results. The economic environment is positive, and the average per capita income is higher, indicating that a better local economic situation can attract many human resources, enterprises, and trade activities, thereby effectively improving the economic benefits of high-tech IDZs. In other words, the better the economic environment of high-tech IDZ, the more conducive to the development of high-tech IDZ, the more complete the economic structure, and the more significant the scale economy effect of the internal industrial chain. Also, the number of talents and the economic efficiency of high-tech IDZ share a significant positive correlation. Accumulating high-quality talents in high-tech IDZs can produce a talent gathering effect, increasing talent integration, thereby enhancing the independent innovation ability of high-tech IDZs. The high-tech IDZ’s regional scale and economic benefits have limited impact and are of little significance. Test results show that the scale of high-tech IDZ has a positive effect on improving the economic efficiency of high-tech IDZ, but the effect is not notable. Instead, if the GDP scale of high-tech IDZ is excessive, immense, its economic efficiency will decline. The capital investment is significantly positively correlated with the economic efficiency of high-tech IDZ. The high-tech IDZ’s technological innovation network with substantial capital investment has a faster flow of elements, stronger scientific research capabilities, and greater competitiveness than other high-tech IDZs, showing great advantages, which can greatly improve the economic efficiency of high-tech IDZ.

**Fig 5:** Regression analysis results of high-tech IDZ’s economic efficiency influencing factors.

### Model performance analysis

Fig 6 shows the comprehensive efficiency results of high-tech IDZs in different provinces and different years. Here, the Data Envelopment Analysis Processing (DEAP) software is utilized, which is a DOS program that runs under the WINDOWS interface. The DEAP software is adopted to calculate and analyze the high-tech IDZs’ comprehensive efficiency, PTE, and scale efficiency. The best performed high-tech IDZ in the Northern region is Taiyuan High-tech IDZ, with an average comprehensive model efficiency of 0.6813; the best performed high-tech IDZ in the Southern region is Xiamen High-tech IDZ, with an average comprehensive model efficiency of 0.9755; the best performed high-tech IDZ in Eastern region is Jiangsu High-tech IDZ, with an average comprehensive model efficiency of 0.91118; the best performed high-tech IDZ in the Western region is Lanzhou High-tech IDZ, with an average comprehensive model efficiency of 0.878. However, the overall efficiency of different high-tech IDZs is more significant than 0.5. Therefore, the results of all models are effective and can reflect the real economic situation. Xiamen High-tech IDZ has focused on developing advantageous industries, attracting many talents through the dual innovation platform, and attracted a large number of enterprises and industries through innovative policies, which is reflected in the results. These are advantages unmatched by other high-tech IDZs. However, in contrast, many cities in Northern China have lower economic indexes. The primary reason is that the Northern region’s economic development is not so strong, and the transportation system is not complete. Therefore, these cities are at a long-term disadvantage in the fierce competition, resulting in slow economic development and low high-tech IDZ economic efficiency. The high-tech IDZ cannot be supported by a strong funding policy so that the economic efficiency is naturally much lower.

RETRACTED

**Fig 6:** Comprehensive efficiency results of high-tech IDZs in different years and different provinces.

### Economic change analysis

Fig 7 shows the economic efficiency results of high-tech IDZs in different provinces and different years. The PTE value of Beijing High-tech IDZ in ten years is 1, and the PTE value of Xiamen, Xi’an, and Urumqi high-tech IDZs is 1 in at least seven years. The average values of PTE of the three high-tech IDZs in Taiyuan, Changsha, and Luoyang rank the bottom three, which are 0.6987, 0.7406, and 0.6595, respectively. The above results show that the TE values of the three high-tech IDZs are relatively poor. The reason is that the capital investment of science and technology is small, and the independent innovation ability is relatively weak.

**Fig 7:** Economic efficiency results of high-tech IDZs in different provinces and different years.

### Scale efficiency analysis

Fig 8 illustrates the scale efficiency results of high-tech IDZs in different provinces and different years. In terms of high-tech IDZ’s scale efficiency, except for Beijing High-tech IDZ with a scale efficiency value of 0.5794, this index of other high-tech IDZs is relatively high. Specifically, Xiamen High-tech IDZs’ scale efficiency is maintained at 1 for more than seven years in 2009–2019, ranking a relatively high position in high-tech IDZs. The average scale efficiency of Hangzhou High-tech IDZ is 0.9839. Compared with the comprehensive efficiency and PTE, its scale efficiency value has been dramatically improved. The high scale efficiency of Hangzhou high-tech IDZ may be due to Hangzhou’s developed logistics industry and excellent business environment. In general, the scale efficiency values of most high-tech IDZs are practical, which also shows that the expansion of high-tech IDZs that the Chinese government has vigorously promoted in recent years has achieved good results.

RETRACTED

**Fig 8:** Scale efficiency results of high-tech IDZs in different provinces and different years.

### Super efficiency analysis

Fig 9 illustrates the super efficiency results of high-tech IDZs in different provinces and different years. Xiamen and Jiangsu high-tech IDZs, located in Southern China, have the highest average super efficiency; the particular values are 1.3519 and 1.2336 on average, while Beijing, Hangzhou, and Luoyang high-tech IDZs are ranked lower, with super-efficiency values of 0.5794, 0.0.5547, and 0.5858 on average. The rapid development of Xiamen’s high-tech IDZ depends on the results of regional management and industrial restructuring. Many high-tech industries have settled in Xiamen, mostly technological enterprises, which directly promote the industrial development of the region. However, due to the rapid development of high-tech industries in Beijing and Hangzhou and the outflow of talents from Beijing in recent years, the development of high-tech industries in these regions has been relatively slow.

**Fig 9:** Super efficiency results of high-tech IDZs in different provinces and different years.

### Regional economy analysis

Fig 10 shows the dynamic efficiency changes of different high-tech IDZs. The Eastern China high-tech IDZ index is as high as 1.017. The primary driving factor is the change in technology, which has increased by 1.7%. The index of the central region is 1.061. This region is significantly better than the Eastern region; the improvement mainly comes from TE and TC, which has increased by 6.1%.

**Fig 10:** Dynamic efficiency changes of high-tech IDZs across China in different years.

Meanwhile, the index of the Northern region is 1.046, which is in the middle reaches, and the index is increased by 4.6%. The Western region index is 1.052, and TC is increased by 0.3%, but TE is dropped by 7.8%. This shows that the high and new technologies in the Western region need further improvements. Except for the Western region, the PTE of other regions is greater than 1, indicating that the high and new technologies in these regions are improving continuously. The above analysis suggests a lot of room for improvement in the regional economy of all regions. Different high-tech IDZs can use their location advantages to form a benign complement and perfection, effectively reducing the differences between regions.

RETRACTED

Fig 11 shows the changes in high-tech IDZs in different years. The differences between high-tech IDZ economies are large in different periods, and the index changes in different periods are also different. Among them, in 2011, 2013, and 2017, the index of high-tech IDZs increased by 7.9%, 18.4%, and 8.3%, respectively; however, in some years, the index declined. Such a decline may be associated with the global economic recession. Overall, the trend is rising, especially the rapid development of the internet economy in recent years has led to the overall economic stability at a relatively high level, which is consistent with the actual economic development. Therefore, the model proposed can predict economic changes well.

**Fig 11:** National high-tech IDZs’ productivity index and decomposition results in different years.

The above analysis reveals that after nearly 30 years of rapid development, China’s high-tech IDZs have made considerable progress, and the comprehensive strength and competitiveness have been significantly improved. However, there are structural problems and uneven development between regions. Therefore, creating a first-class business environment is necessary to optimize the economic environment and reduce the number of enterprises in high-tech IDZs. The stock of human capital should be increased to enhance the innovative capabilities of high-tech IDZs. The accumulation of talents should be strengthened, the investment in science and technology should be increased, and the innovation ability of high-tech IDZs should be enhanced.

## Discussion and analysis

The above analysis reveals that after nearly 30 years of rapid development, China’s high-tech IDZs have made considerable progress, and their overall strength and competitiveness have improved significantly. However, there are structural and regional unbalances among the IDZs across China. Thus, the specific measures to improve the economic efficiency of high-tech IDZs are explored from the directions of the economic environment, the number of talents, investment in science and technology, and the scale of high-tech IDZs. (1) A first-class business environment shall be created to optimize the economic environment. The problems in the business environment of the high-tech IDZs are reflected in the cost of business management in each high-tech IDZ and the efficiency of each link. (2) The operating and management costs of enterprises in high-tech IDZs shall be reduced, and the financing environment for enterprises in high-tech IDZs shall be improved. Financial institutions are encouraged to strengthen the critical assistance to high-tech IDZs in underdeveloped areas and implement preferential measures, such as classified assistance to high-tech enterprises and lower loan interest rates. (3) The efficiency of enterprises in the high-tech IDZs shall be improved. A sound business environment can promote enterprise development and improve the efficiency of enterprises so that some of the functions of the high-tech IDZs can be reflected, such as the establishment of information exchange platforms, regional collaborative development work, enterprise incubator, and innovation driving ability. This is a benign interaction, a mutual benefit, and a win-win situation, which is precisely the long-term mechanism that genuinely promotes the development of high-tech IDZs. (4) The stock of human capital shall be increased to strengthen the accumulation of talents. IDZs should also cooperate extensively with the research institutes and universities, allowing talents from these institutions to practice in enterprises and cultivating an “ecological chain” in which enterprises and these institutions can achieve a win-win situation. The proposed model can reduce the government’s management expenditure and effectively help the government organs analyze the economic conditions of the country and different provinces, which is very important for the implementation of policies. However, in practical applications, professional technicians are required for analysis, resulting in more demand for talents in mathematical statistics and computer science. Due to the low management cost of government organs, many talents are unwilling to engage in such technical analysis work. This is the principal problem that may occur during the promotion of this model. Nevertheless, such talents can be attracted by appropriately increasing the welfare of enterprises and individuals.

RETRACTED

## Conclusions

Based on previous research, factors that affect economic efficiency are theoretically analyzed, the characteristics of different high-tech IDZs are clarified, and the economic efficiency is divided using ML-based data processing methods. The economic changes in different regions are analyzed from four dimensions: economic structure, number of talents, capital input, and regional scale. Finally, a specific economic analysis theoretical model is derived. Cities with higher overall efficiency are in the northern and the eastern regions. The high-tech IDZ index in the eastern region is 1.017, whose contributing factor is the technological change that has increased by 1.7%. The high-tech IDZ index in the central region is 1.061, which is superior to the eastern region. The contributing factors include technical efficiency and changes, which have increased by 6.1%.

In comparison, the high-tech IDZ index in the northern region is 1.046, which is in the relatively middle reaches and has increased by 4.6%. Finally, the high-tech IDZ index in the western region is 1.052, in which the technical changes have increased by 0.3%, but the efficiency has decreased by 7.8%. The above results show that the high and new technology in the western region can be further improved. The index of high-tech development IDZs is high. A decreasing trend appears in individual years, which may be associated with the global economic recession. However, the overall trend is increasing. The rapid development of the internet economy in recent years has led to high overall economic stability, which is consistent with actual economic development. Increasing the proportion of the secondary industry, the number of employees and the funding investment will effectively improve the economic efficiency of high-tech IDZs. The above results also explain that it is necessary to continue building a first-class business environment, increase talent and capital storage, promote high-tech IDZ expansion, and develop industrial clusters. Although a suitable economic analysis model has been established, and different economic data are analyzed profoundly, several shortcomings are found. First, different national high-tech IDZs in China have been analyzed; however, these samples have not been expanded to high-tech IDZs in other countries. The problems in the development of China’s high-tech IDZs can be found in comparison with developed countries. Second, the research period is relatively short. The high-tech IDZ’s influencing factors should be refined continuously, such as which industries and indexes will affect the scale of industrial development in the high-tech IDZs, thereby comprehensively analyzing the problems existing in the economic development of high-tech IDZs. In the future, the above two aspects will be analyzed profoundly to continuously improve the model proposed and provide better research ideas for the economic development of high-tech IDZs.

## Supporting information

S1 Data (XLSX)
